# Research on Students' Mental Health Based on Data Mining Algorithms

**DOI:** 10.1155/2021/1382559

**Published:** 2021-10-25

**Authors:** Mengjun Luo

**Affiliations:** College of Preschool Education and Humanities, Dongguan Vocational and Technical College, Dongguan, Guangdong 523808, China

## Abstract

With the diversification and rapid development of society, people's living conditions, learning and friendship conditions, and employment conditions are facing increasing pressure, which greatly challenges people's psychological endurance. Therefore, strengthening the mental health education of students has become an urgent need of society and a hot issue of common concern. In order to solve the problems of high misjudgment rate and low work efficiency in the current mental health intelligence evaluation process, a mental health intelligence evaluation system based on a joint optimization algorithm is proposed. The joint optimization algorithm consists of an improved decision tree algorithm and an improved ANN algorithm. First, analyze the current research status of mental health intelligence evaluation, and construct the framework of mental health intelligence evaluation system; then collect mental health intelligence evaluation data based on data mining, use joint learning algorithm to analyze and classify mental health intelligence evaluation data, and obtain mental health intelligence evaluation results. Finally, through specific simulation experiments, the feasibility and superiority of the mental health intelligent evaluation system are analyzed. The results show that the system in the article overcomes the shortcomings of the existing mental health intelligence evaluation system, improves the accuracy of mental health intelligence evaluation, and improves the efficiency of mental health intelligence evaluation. It has good system stability and can meet the actual current situation, which are requirements for mental health intelligence evaluation.

## 1. Introduction

Due to the rapid development of modern society, people's pressure to survive has also risen. The rising pressure of social competition [1, 2] has caused more and more people to have psychological problems such as emotions and behaviors. Every year, psychological barriers [3] and even suffering appear. The number of mentally ill people began to grow substantially. Resolving people's psychological problems [4] caused by various factors has become the most important work. The directions that need to be studied are how to provide people with mental health services [5] and improve the results of mental health work [6]. In response to the above problems, it is necessary to use innovative ideas and concepts, combined with modern technology and information technology, to build a mental health intelligent evaluation system [7] to improve the scientific level of mental work. Some scholars [8–10] have built a mental health service system for the elderly based on the internet technology, and some scholars have built an automatic evaluation system for users' mental health in online forums based on multifeature fusion. Improving users' mental health has improved the data collection and data collection of mental health. Regarding its management, its function is too one-sided, and its applicability is weak. Traditional mental health assessment methods [11–14] are mostly carried out in the form of scales or questionnaires. There will be certain limitations in terms of survey objects and the accuracy of survey results. With the rise of the Internet technology, the application of network technology to mental health assessment has become a new phenomenon. The tendency of survey respondents to self-assess in a more concealed environment can reduce their psychological pressure.

Popular internet software will record user status to varying degrees. It can be seen that the Internet evaluation system is a highly applicable way of evaluating the mental health of college students [15]. Papineni et al. [16] proposed an automatic evaluation method for online forum users' mental health, designed an evaluation framework, hierarchically analyzed the data reflecting the user's mental health, and used different methods to fuse user psychological data to obtain a more comprehensive evaluation method. The system takes a long time; Soet [17] designed a college student mental health consulting service system based on the web, carefully analyzed user needs, and divided the system into different functional categories to build the entire mental health consulting service system to help users better provide psychological services, but the recall rate is not high. David et al. [18] selected the research object for the elderly and used different theoretical models for this group to conduct mental health tests, evaluate the advantages and disadvantages of different models, and integrate the advantages of various theoretical models. A mental health assessment method [19] is proposed, but the accuracy rate needs to be improved. Yang et al. [20] research object is also the elderly, and they analyzed the system requirements, designing an overall mental health assessment framework, and analyzed them one by one, but the system is efficient in operation room for improvement. With the continuous improvement of the ability to collect, analyze, and process data in the era of big data, it is no longer necessary to use paper questionnaires to sample data. People can accurately capture various data dynamics through computers combined with big data technology. In past research, schools mainly used paper questionnaires to measure students' mental health [21]. This method consumes manpower and material resources and is costly. Using big data technology, mental health assessment can be extended to a larger scope. Students use the internet to generate massive amounts of big data and use big data technology [22] to build a mental health evaluation system, which can fully grasp the psychological dynamics of students, combined with the establishment of mental health scales, and can more accurately predict the mental health of students.

The application of machine learning [23–25] in the field of mental health has gradually become an important development trend. Machine learning is a process of automatically analyzing or predicting new and unknown data by discovering the laws of a large amount of existing data and information. Tom gave a formal definition of machine learning: assume that performance is used to evaluate the performance of a computer program on a certain task if the program obtains performance improvement on the task by using experience. The currently available data types for machine learning are (1) text data [26]. Its sources include social media, clinical assessments and records, electronic health records, and diaries. In particular, social media can provide a large amount of data reflecting individual psychological and behavioral traces, which has higher ecological validity. At present, it mainly focuses on the prediction of suicide risk, the analysis of personality traits, the prediction of mental health status, and subjective well-being. (2) Survey data [27] is commonly used is the combination of demographic variables, psychological scales, and publicly authoritative statistical data to predict and diagnose mental illnesses such as personality types and mental disorders. (3) Brain imaging data [28]: the detection of traditional brain imaging data relies too much on expert judgment, is time-consuming and laborious, and has a high misdiagnosis or missed diagnosis rate. The accuracy of automatic classification using machine learning is better than expert judgment. Currently, it is commonly used in the prediction of cognition, memory, emotions, and addictive behaviors. (4) Behavioral and physiological data [29]: it mainly comes from eye-tracking, portable mobile devices, multichannel physiological recorders, and expression analysis systems. Machine learning algorithms are divided into three categories: (1) supervised learning [30, 31]; (2) semisupervised learning [32]; (3) unsupervised learning [33]. Supervised learning is to obtain the relationship between data with features and labels through training to judge new data. Use labeled data to train the model. The model can predict the label of new data. For example, [34] the machine learning model can automatically identify based on the brain imaging data of traumatic brain injury patients and normal individuals to distinguish individual illnesses. Unsupervised learning is to discover the relationship between unfeatured and labeled data through training to judge new data. In many cases, labeled data sets may be difficult to obtain, so the model's predictive ability can be enhanced by using unlabeled data, but it should be understood that no algorithm can solve every problem well. Hence, it is necessary to compare multiple algorithms to determine which algorithm is most suitable for a particular data set and task to be solved. Commonly used machine learning algorithms include decision trees [35], naive Bayes [36], support vector machines [37], K-nearest neighbors [38], logistic regression [39], multilayer perceptions [39], random forests [40], and K-Means [41].

To improve the effectiveness of mental health intelligence evaluation, this paper proposes a mental health intelligent evaluation system based on data mining, which can effectively promote system information management, solve problems such as the old system resources, make perfect use of internet advantages, create a new internet environment, and effectively solve the psychological problems of contemporary people.

## 2. Related Work

The goal of psychology [42] is to describe, explain, predict, and control behavior. At present, most psychological research focuses on describing and explaining the relationship between variables. Research that can truly achieve the prediction goal is not common, and traditional psychological research [43] is due to the small sample size. The results of some studies are contradictory and uncertain due to low data quality and lack of covariate information. And, the significance test based on *p* value faces a crisis of duplication, that is, the irreproducibility of research results. Strict and systematic use of machine learning cross-validation technology [44] can provide great potential for realizing the reproducibility of psychological research. Technology-based machine learning can construct learning models from massive amounts of data, more accurately identify the underlying laws of the data, and have stronger generalization capabilities. The model can be applied to different samples or groups, thereby minimizing prediction errors to make more accurate results.

Many researchers try to use machine learning to predict complex psychological problems of individuals, such as predicting stress disorders and anxiety disorders. The research of Tian et al. [45] and Zhu et al. [46] found that only the effective features that can predict the possibility of suicide can reach thousands. They use a multilayer perceptron algorithm to build a suicide recognizer for Weibo social media to evaluate the suicide of Weibo users in real time. As regards possibility, the prediction accuracy rate can reach about 94%. Carpenter [47] used preschool psychiatric assessment data and machine learning to assess the risk of anxiety in children aged 2 to 5 years, and their prediction accuracy for generalized anxiety disorder and separation anxiety disorder was as high as 90%.

Moreover, machine learning usually does not make assumptions or establish relationships between independent variables and dependent variables. It usually makes judgments among all possible independent variables, gives prediction results, and outputs important independent variables. Walsh [48] used the random forest model to predict future suicide behaviors of suicide attempted patients and normal subjects. The independent variables used include demographic variables, medical records, and socioeconomic status, and the accuracy of the predictive indicators can reach about 89%. Moreover, the long-term prediction cycle is the most important predictor for those who have attempted suicide in the history of hospital visits; in the short-term prediction cycle, dependence on addictive drugs is an important predictor. The type indicates that the activation degree of the amygdala and the hippocampus during the cognitive reassessment task and the amygdala gray matter volume have a good predictive ability for borderline personality disorder, and its accuracy and sensitivity can reach more than 70%. Such prediction results are correct. The development and selection of personalized mental interventions are crucial. In order to enable people to have an accurate understanding of their mental health, and at the same time to promote the scientific and informatization of mental health guidance, this paper constructs a mental health intelligent evaluation system based on a decision tree algorithm, using scientific mental health evaluation. The tool provides a comprehensive and objective reflection of the user's mental health. The overall structure of the system is shown in Figure 1.

## 3. Methodology

### 3.1. Improved Decision Tree Algorithm

#### 3.1.1. Entropy for Preprocessing

The client software of this system uses the method of psychological evaluation data mining to realize the evaluation results, processes the obtained user evaluation result data and establishes a database, analyzes the evaluation results through the decision tree algorithm, and obtains evaluation. Psychological assessment data mining includes extracting data from the database, cleaning the data, selecting the mining model, and outputting the results. The complete data mining process is shown in Figure 2. In this paper, the system uses the user's answer results to establish an initial data set. After preprocessing data integration, data extraction, data cleansing, and data conversion, a mental health assessment data set to be mined is obtained. The decision tree algorithm is applied in the mining process. The data classification is obtained through the mining results, thereby obtaining the specific classification of the user's mental health status.

The decision tree algorithm is an inductive learning algorithm, a classification rule obtained by inducing a set of chaotic examples based on examples. The decision tree mainly includes two steps when processing the classification problem. The first is to generate a decision tree classification model through the learning and training set; the second is to classify unknown types of samples through the model. In the classification process of a certain sample type, the root node is the starting point, a leaf node is an endpoint, and the sample attributes are gradually tested in the downward direction of the branch. In this paper, the C4.5 decision tree algorithm is applied, and the splitting index is the information gain rate, which solves the problem of biasing the selection of multiple attributes when using information gain to select test attributes. The definition formula of information gain rate is

(1) $$\begin{array}{c} \text{gain ratio}=\frac{\text{Gain}\left(S,A\right)}{\text{Split Information}\left(S,A\right)}. \end{array}$$

Gain(*S*, *A*) is the information gain of the attribute *A* and SplitInformation(*S*, *A*) is the breadth and uniformity of splitting the sample set *S* according to the attribute *A*.

The decision tree C4.5 algorithm is used to classify the mental health intelligence assessment data to provide data support for the system in this paper.

(2) $$\begin{array}{c} \text{SplitInformation}\left(S,A\right)=-\overset{n}{\underset{i=1}{\sum }}\frac{\left|S_{i}\right|}{\left|S\right|}\log_{2}\left(\frac{\left|S_{i}\right|}{\left|S\right|}\right). \end{array}$$

In the process of decision tree generation, the most important thing is to determine the split target. In order to determine the splitting index in the C4.5 algorithm, it is necessary to compare the size of the attribute information gain rate in each training sample data and select the attribute with the largest information gain rate and higher than or equal to the average value of all attributes as a branch node of the decision tree for the existence of continuous descriptive attributes; the continuity needs to be divided to obtain a discrete set of intervals. Discretization methods include the following:

1. Discretize the continuity attribute *A* of the continuous interval value. The continuity attribute values are arranged in the training set *S* samples in ascending order, and the minimum and maximum values in the interval are assigned to MIN and MAX, respectively, to obtain the value sequence of the attribute value which is {*A*_1_, *A*_2_,…, *A*_*n*_}.
2. Suppose *A*_*i*_ is the equal division point. If there are *N* equal division points in the interval [MIN, MAX], calculate in order, and the formula for the *i*-th equal division point is *A*_*i*_=MIN+*i∗*(MAX − MIN), where *i*=1,2,…, *N*.
3. Calculate the information gain values in the interval values [MIN, *A*_*i*_] and [*A*_*i*_, MAX], respectively, and there is a total of *N* − 1 dividing points for comparison.
4. Suppose the segmentation threshold of continuity attribute *A* is the segmentation point with the largest information gain rate *A*_*k*_, divide the data set based on this, and set the attribute value in [MIN, *A*_*k*_] and [*A*_*k*_, MAX].

According to the above discretization method, the information gain rate of all attributes in the candidate attribute set is solved, and the test attribute is the attribute with the largest information gain rate. Use all possible values in the sample set to divide the sample to obtain several subsample sets. Use the same method to continue to divide all the subsample sets. Until it cannot be divided, the decision tree is generated. When using the C4.5 algorithm to generate a decision tree, the selected target class affects the determination of each class. When evaluating the decision tree, information entropy needs to be used to obtain

(3) $$\begin{array}{c} S=-\underset{i}{\sum }\left(P_{i}*\;\log_{2}P_{i}\right). \end{array}$$

Information gain is the effective reduction of information entropy. According to information entropy, the variable level used for classification can be determined. If there are two classes, class *A* and class *B*, in the training set *S*, and they, respectively, include *x* and *y* records belonging to class *A* and class *B*, then the formula for determining the total amount of information for a certain record in the training set *S* is

(4) $$\begin{array}{c} \text{Info}\left(s\right)=\text{Info}\left(s_{a},S_{b}\right)=-\left(\frac{x}{x+y}\right)\cdot \;\log\frac{x}{x+y}+\frac{y}{x+y}\cdot \;\log\frac{y}{x+y}. \end{array}$$

Suppose variable *C* is the root node of the decision tree, and the subclasses of training set *S* are divided into {*S*_1_, *S*_2_,…,  *S*_*k*_}; then *S*_*i*_(*i*=1,  2,…,  *k*) includes *X*_*i*_, *Y*_*i*_ records that belong to class *A* and class *B*, respectively. Get the information volume formula classified in all subcategories:

(5) $$\begin{array}{c} \text{Info}\left(C,S\right)=\overset{k}{\underset{i=1}{\sum }}\frac{x_{i}+y_{i}}{x+y}\text{Info}\left(S_{iA},S_{iB}\right). \end{array}$$

Suppose variable *C* is the classification node of the decision tree, and its information increment value is the largest among all variable information increment values. Then the information increment formula of variable *C* is

(6) $$\begin{array}{c} \text{Gain}\left(C\right)=\text{Info}\left(S\right)-\text{Info}\left(A,S\right). \end{array}$$

Then the information gain function is defined as

(7) $$\begin{array}{c} \text{Gain}\left(D,C\right)=\text{Info}\left(S\right)-\text{Info}\left(D,S\right),\\ \text{Info}\left(S\right)=-\left(P_{1}*\;\log\;P_{1}+\cdots +P_{k}*\;\log\;P_{k}\right),\\ \text{Info}\left(D,S\right)=\overset{n}{\underset{i=1}{\sum }}\frac{\left|S_{i}\right|}{\left|S\right|}\text{Info}\left(S_{i}\right). \end{array}$$

#### 3.1.2. Improved Decision Tree

From the basic principle of the C4.5 algorithm, it can be known that the selection of attributes when generating a decision tree is based on the principle of information theory. Since the calculation of the information gain rate formula involves multiple logarithmic function operations, this requires that the library function is called multiple times during calculation, which greatly increases the calculation time. In response to this problem, an improved method for calculating the information gain rate is proposed; that is, the mathematical Taylor formula and McLaughlin's formula are used to simplify the calculation of the information gain rate of the C4.5 algorithm, which greatly reduces the calculation of the algorithm. The improved C4.5 algorithm is named TAM-C4.5 algorithm.

Since the derivative of ln(*x*) at *x*=0 is meaningless, and the commonly used probability value range in the calculation formula of information gain rate is between [0,1], this paper chooses the Maclaurin formula of ln(*x*+1) which improves the calculation formula of information gain rate in traditional C4.5, as the formula

(8) $$\begin{array}{c} \ln\left(x+1\right)\approx \;x-\frac{1}{2}x^{2}+\frac{1}{3}x^{3}+\cdots +{\left(-1\right)}^{n-1}x^{n},\\ \ln\left(x\right)\approx \;\left(x-1\right)-\frac{1}{2}{\left(x-1\right)}^{2}+\frac{1}{3}{\left(x-1\right)}^{3}+\cdots +{\left(-1\right)}^{n-1}{\left(x-1\right)}^{n}. \end{array}$$

When *x* ∈ (0,1), the formula will become as follows:

(9) $$\begin{array}{c} \ln\left(x\right)\approx \;\left(x-1\right)-\frac{1}{2}{\left(x-1\right)}^{2}+\frac{1}{3}{\left(x-1\right)}^{3}. \end{array}$$

Through the above approximate simplification, it is possible to convert logarithmic operations into nonlogarithmic operations, and the abovementioned conversion characteristics can be used to eliminate complex logarithmic operations in the information gain rate formula, so as to simplify the calculation formula and improve the efficiency of tree construction.

The conversion formula of category information entropy is as follows:

(10) $$\begin{array}{c} {\text{Info}}^{\prime }\left(S\right)=\;-\overset{m}{\underset{i=1}{\sum }}\frac{S_{i}}{S}\log_{2}\frac{S_{i}}{S}. \end{array}$$

Similarly, the conversion formula of conditional information entropy and split information entropy is as follows:

(11) $$\begin{array}{c} {\text{Info}}_{A}^{\prime }\left(S\right)=\;-\frac{1}{\ln\left(2s\right)}\overset{k}{\underset{j=1}{\sum }}\overset{m}{\underset{i=1}{\sum }}\left[\frac{s_{ij}\left(s_{ij}-s_{j}\right)\left(11s_{j}^{2}+2s_{ij}^{2}-7s_{ij}s_{j}\right)}{6s_{j}^{2}}\right],\\ {\text{Info}}^{\prime }\left(A\right)=\;-\frac{1}{\ln\left(2s\right)}\overset{k}{\underset{j=1}{\sum }}\left[\frac{s_{j}\left(s_{j}-s\right)\left(11s^{2}+2s_{j}^{2}-7s_{j}s\right)}{6s^{2}}\right]. \end{array}$$

Therefore, the formula for calculating the information gain rate after conversion is as follows:

(12) $$\begin{array}{c} \text{Gain}-{\text{Ratio}}^{\prime }\left(A\right)=\frac{{\text{Info}}^{\prime }\left(S\right)-{\text{Info}}_{A}^{\prime }\left(S\right)}{{\text{Info}}^{\prime }\left(A\right)}. \end{array}$$

Analyzing the improved calculation formula shows that the category information entropy is the same every time the information gain rate value of the condition attribute is calculated. Since 1/ln(2*s*) is omitted in each part of the simplified formula in this article, in order to ensure the classification accuracy of the algorithm, this article is calculating the category conditional entropy, the improved formula is used to try to ensure that the order of the information gain rate of each condition attribute is not changed, and the classification accuracy is not affected. The traditional C4.5 algorithm needs to call a function to perform a large number of logarithmic function operations. The improved algorithm proposed in this paper only needs a simple four-mixed operation, which eliminates the frequently called logarithmic operation in the information gain rate calculation formula, and the system operation speed is greatly improved.

### 3.2. Improved ANN Algorithm

#### 3.2.1. ANN for Prediction

An ANN is a structure and calculation model that imitates a biological neural network. It is usually used to estimate or approximate a function. The neural network is mainly composed of the input layer, hidden layer, and output layer. In practice, each neuron in the network's input layer represents a feature, and the number of neurons in the output layer is one. If the Softmax classifier as shown in Figure 3 is used, the number of output neurons is two, a multiclassification problem. The number of hidden layers and hidden layer neurons is manually set.  Figure 4 shows a basic neural network model.

The MP neuron model receives input signals from other neurons, and the connections are transmitted. Then the total input received by the neuron is compared with the neuron's threshold, and after the activation function is processed, the neuron's output is generated.

Ideally, the form of the activation function should be a step function (that is, the modified linear unit ReLU). There are two output types: 0 or 1. 0 means that the neuron is not excited, and 1 means that the neuron is excited. But the step function is not smooth and discontinuous, so the activation function usually chooses the sigmoid function.

It can be seen from the function image that the value range of the function is (0,1). That is, the function value falls between 0 and 1. The property of the sigmoid function is that it can compress the input value that changes in a larger range into the (0,1) interval, so it is also called a squashing function. By connecting many neural units according to a certain level, a neural network is obtained.

#### 3.2.2. The Cross-Entropy Cost Function to Optimize Backpropagation

When using this method, the real output *y* should be transformed by the Softmax function first and then calculated in the substitution cost function. The calculation formula of the softmax function and classification cross-entropy is as follows:

(13) $$\begin{array}{c} y_{\text{out}}^{i}=\text{softmax}\left(y_{k}^{i}\right)=\frac{e^{y_{k}^{i}}}{\sum_{q=1}^{k}e^{y_{k}^{i}}},\\ J\left(\theta \right)=-\overset{m}{\underset{i=1}{\sum }}\overset{k}{\underset{k=1}{\sum }}y_{k}^{i}\;\ln\;y_{\text{out}}^{i}+\frac{\lambda }{Z_{m}}\overset{s}{\underset{i=1}{\sum }}\overset{sl+1}{\underset{j=1}{\sum }}\theta_{j.i}^{{\left(i\right)}^{2}}. \end{array}$$

When we improve the classification loss, we need to optimize the gradient of a step size through gradient descent. At this time, we require loss to give the partial derivative of each weight matrix and then apply the chain rule. Then the first step in this process is to derive the softmax.

Calculate the error for the output *y* that the Softmax function has not transformed; that is, find the derivative of *a*. According to the chain rule, it can be transformed into an error function. The derivative of the output after the transformation of the softmax function is multiplied by the derivative of the output after the transformation of the SoftMax function, and the calculation formula for the derivative of *a* is as follows:

(14) $$\begin{array}{c} \frac{\partial J\left(\theta \right)}{\partial a}=\frac{\partial J\left(\theta \right)}{\partial s}\cdot \frac{\partial s}{\partial a}. \end{array}$$

Among them, the formula for the loss function to derive the softmax layer is

(15) $$\begin{array}{c} \frac{\partial J\left(\theta \right)}{\partial s}=\;-\overset{K}{\underset{k=1}{\sum }}y_{k}\cdot \frac{1}{S_{k}},\\ S_{k}=\frac{e^{a_{k}^{3}}}{e^{a_{k}^{1}}+e^{a_{k}^{2}}+e^{a_{k}^{3}}+\cdots +e^{a_{k}^{n}}}, \end{array}$$

where *y* is the expected output value of the  *k*-th neuron and *s*_*K*_ is the output of the *k*-th neuron transformed by the softmax function, namely, *y*_out_.

#### 3.2.3. Improved ANN Algorithm

Based on ANN's three-layer perceptron and nonlinear optimization capability, it can approximate any nonlinear function. However, ANN also has areas that need to be improved. (1) There are many times of training, and the convergence speed is relatively slow. The ANN algorithm also needs a lot of learning and training to converge for simple and common problems. For more complex problems, the training time will be longer. Using the gradient descent method to minimize the loss function will inevitably cause jagged images, resulting in low algorithm efficiency. In order to better solve this problem and improve the convergence speed of the ANN network, the momentum term can be appropriately increased, the error function can be improved, the learning rate can be adaptively changed, and the steepness factor can be used. (2) It is easy to fall into the local optimum, and the global optimum cannot be guaranteed. Because the backpropagation algorithm uses the gradient descent method, the weight space is a parabola with a minimum point, and there are multiple minimum points. Therefore, different training starting points will result in no optimal solution.

At present, there are many researches on ANN improvement. The more commonly used optimization algorithms are additional momentum algorithm, variable algorithm, adaptive learning rate method, RPROP method, conjugate gradient algorithm, Newton algorithm, Levenberg–Marquardt algorithm, etc. LM algorithm has the fastest convergence speed and the best robustness among the above algorithms.

In Newtonian algorithms, if Hessian matrix is not a positive definite matrix, then the Newtonian direction may point to a local optimum. This phenomenon can be solved by adding a positive definite matrix to Hessian matrix. LM algorithm is a combination of gradient descent method and Gauss–Newton method. It also has local convergence and global characteristics of gradient descent method. LM algorithm is also more stable and converges faster than gradient method. In ANN, the loss function ist

(16) $$\begin{array}{c} E\left(x\right)=\frac{1}{2}\overset{n}{\underset{i=1}{\sum }}{\left[d\left(i\right)-y\left(i\right)\right]}^{2}. \end{array}$$

The updated weight is calculated as follows:

(17) $$\begin{array}{c} x^{\left(k+1\right)}=x^{\left(k\right)}+∆x. \end{array}$$

With Newton's algorithm, the amount of change is calculated as follows:

(18) $$\begin{array}{c} \Delta x=-\frac{\nabla E\left(x\right)}{\nabla^{2}E\left(x\right)}. \end{array}$$

Approximate them so that all Hessian matrices are invertible as follows:

(19) $$\begin{array}{c} \nabla E\left(x\right)=J^{T}\left(x\right)e\left(x\right). \end{array}$$

LM algorithm is able to improve the Gauss–Newton method, and the improved weight and threshold adjustment rule is calculated as follows:

(20) $$\begin{array}{c} ∆x=-{\left[J^{T}\left(x\right)J\left(x\right)+µI\right]}^{-1}J\left(x\right)E\left(x\right). \end{array}$$

## 4. Experiments and Discussion

### 4.1. Data Set

This experiment selects Student-Life and Reach Out online forum post data as the data source. The Student-Life data set is a data set researched by Dartmouth College. It records 49 students' psychological perception data for ten consecutive weeks, including academic data, online psychological test data, and questionnaire survey data. Reach Out online forum posts include user posting information, posting time, likes and views, etc. Select 5 million data points from each of the two data sets for a total of 10 million data sets. The data set is equally divided into 10 equal parts, of which six parts are used for neural network model training and four parts are used for experimental testing.

### 4.2. Evaluation Metric

To show the superiority of our proposed method, four evaluation metrics are used to evaluate each algorithm, named MSE, MAE, RMSE, and MAPE.

The MAE of normalized data is given by the following:

(21) $$\begin{array}{c} \text{MAE}=\frac{1}{n}\overset{n}{\underset{i=1}{\sum }}\left|P_{i}-T_{i}\right|. \end{array}$$

The MSE of prediction is as follows:

(22) $$\begin{array}{c} \text{MSE}=\frac{1}{n}\overset{n}{\underset{i=1}{\sum }}{\left(P_{i}-T_{i}\right)}^{2}. \end{array}$$

The equation of MAPE is as follows:

(23) $$\begin{array}{c} \text{MAPE}=\frac{1}{n}\overset{n}{\underset{i=1}{\sum }}\left|\frac{P_{i}-T_{i}}{T_{i}}\right|. \end{array}$$

The RMSE is described as follows:

(24) $$\begin{array}{c} \text{RMSE}=\sqrt{\frac{1}{n}\overset{n}{\underset{i=1}{\sum }}{\left(P_{i}-T_{i}\right)}^{2}}. \end{array}$$

### 4.3. Comparison with Other Methods

Select the following experimental indicators for verification and analysis. Feature fusion accuracy rate: the accuracy of feature fusion is directly related to the accuracy of the system evaluation results, so this indicator is selected for analysis. System recall rate: the recall rate generally refers to the recall rate, which refers to the ratio of the information obtained from the system query to the total amount of system information. The system recall rate is tested to verify the performance of the system in this article. Running time: time consumption is usually an important indicator of system performance. The comparison results of feature fusion accuracy are shown in Figure 5.

According to the comparison curve of the feature fusion accuracy rate of different systems in Figure 5, the system's accuracy rate in this paper is always the highest, with an average value of about 90%. Among the other three results, [16] has higher feature fusion accuracy, the highest rate can reach 80%, and the accuracy rate of [17] and [18] is low. It can be seen that this paper is based on a neural network for multifeature fusion, fully utilizes the ability of a neural network to process data in parallel, and obtains the feature fusion effect with higher accuracy. The higher the system recall rate, the higher the recall rate, and the superior system performance can be obtained.  Table 1 and Figure 6 show the comparison results of the recall rate between the system in this paper and the system in [16], [17], and [18].

By analyzing the table data, it can be found that the system in this paper has a high data recall rate. Under different test data volume conditions, the recall rate is high, and it is much higher than the results of other documents. The system in this paper has certain advantages. By analyzing Figure 6, we can see that the data processing time of the system in this paper has been lower than the other two systems. As the amount of data increases, the data processing time of the three systems has changed. The data processing time of comparison system 1 and comparison system 2 has increased sharply with the increase in the amount of information, and the fluctuation range is large, and the stability is poor. The system's data in this article increase in processing time is small, the curve is smoother, and the stability is good. After the data volume reaches 5 × 10 GB, the data processing time gradually stabilizes, proving that the system in this paper has high data processing efficiency and strong stability.

Table 2 shows the values of each metric obtained in 10 experiments for each algorithm. To further demonstrate the superiority of our proposed algorithm, the histogram is used to compare the average of ten experiments. It is not difficult to find that the error of our proposed algorithm is much smaller than the other two methods. In addition, the box plot shown in Figure 7 is used here to compare the robustness of various algorithms, and we use MSE as the comparison standard. The information entropy method combined with neural networks has far better immunity to extreme and outlier data than other methods.

### 4.4. Evaluation on Joint Optimization

As mentioned before, the proposed joint optimization model consisted of the improved decision network and the improved ANN. To verify the effectiveness of this joint model, the comparative experiment based on the single improved model is conducted, and the result is shown in Figure 8. IDT is improved decision tree. IANN is improved artificial neural network.

It can be seen from the figure that the joint optimization model can obtain the best performance, with the lowest error index and the highest accuracy index. Its performance is better than any single improved model, which verifies the correctness and reliability of the joint optimization model proposed in this paper. At the same time, it can be seen that, compared to the IDT model, the performance of IANN is better, but it is still lower than the joint optimization model.

In addition, this paper uses the corresponding algorithm to improve the original decision tree and ANN. In order to verify the effectiveness of this improvement measure, a comparative experiment was also carried out, and the experimental results are shown in Figures 9 and 10. DT is original decision tree.

It can be seen that, compared with the initial decision tree algorithm and ANN algorithm, after introducing the information entropy improvement algorithm and the LM algorithm to improve the two, respectively, the performance can be effectively improved. The error index shows a downward trend, while the accuracy rate shows an upward trend, which proves the effectiveness and correctness of these two improvement measures.

## 5. Conclusions and Outlook

In order to improve the effectiveness of mental health intelligence evaluation, this paper constructs a mental health intelligent evaluation system based on the joint optimization model, which consists of the improved decision tree algorithm and the improved ANN. The proposed model can fully help users understand their mental health, solve their psychological problems, and enhance self-awareness. In order to make the system of this article more functional and have better development, it is also necessary to improve the analysis of the system evaluation results, improve the system data loss during a power failure, increase the data backup and recording functions of the system, and solve the problem of waste of storage space—more perfect the function of this text system.

This article has conducted in-depth research on students' mental state perception based on network behavior data and has achieved certain results. However, there is still a lot of work that is not perfect and needs further discussion and research. The future research work will be from the following aspects: (1) the data source is not wide enough. This article only uses the network behavior data in the student's on-campus behavior data, which does not fully represent the student's behavior data. Therefore, the next step is to focus on adding other on-campus network behavior data to the network behavior data. Behavioral data, such as library borrowing records and meal card consumption flow records, are used to construct a perceptual model of students' mental state. (2) There is not enough feature dimensions. The next step will be to explore new feature dimension construction methods. The currently used feature dimension data is only constructed with two indicators of regularity and dependence. In the future, more intermediate variables based on network behavior data will be explored. The existence continuously enriches the feature dimension of the sample data set. (3) The scope of model consideration is not large enough. The model used in this article is only two classification models in machine learning, and the current more popular deep learning model is not used. The next step will be to use the network structure model of deep learning to conduct model experiments and compare the performance of the authors' model.

## Figures and Tables

**Figure 1:** Overall structure of the system.

**Figure 2:** Complete data mining process based on decision tree.

**Figure 3:** The structure of Softmax classifier.

**Figure 4:** The structure of ANN.

**Figure 5:** The comparison results of feature fusion accuracy.

**Figure 6:** Comparison of three systems. (a) Recall. (b) Time consumption.

**Figure 7:** Comparison of different evaluation metrics with different methods. (a) Four metrics. (b) Box plot.

**Figure 8:** Comparison of joint optimization and single improve network. (a) Four metrics. (b) Accuracy.

**Figure 9:** Comparison of IDT and DT. (a) Four metrics. (b) Accuracy.

**Figure 10:** Comparison of IANN and ANN. (a) Four metrics. (b) Accuracy.

**Table 1:** Comparison results of recall rate.

Test numbers	Proposed (%)	Literature [16] (%)	Literature [17] (%)	Literature [18] (%)
100	95	85	62	59
200	96	83	63	58
300	93	81	67	59
400	94	82	65	54

**Table 2:** Comparison of different metrics of different method.

No. 1	Proposed	Literature [16]	Literature [17]	Literature [18]

MAE	4.86*E* + 01	1.51*E* + 02	5.36*E* + 01	3.81*E* + 03
MSE	4.71*E* + 04	8.50*E* + 04	8.98*E* + 03	1.64*E* + 07
RMSE	2.17*E* + 02	2.92*E* + 02	9.48*E* + 01	4.05*E* + 03
MAPE	2.93*E* − 02	4.10*E* − 02	1.63*E* − 02	1.76*E* + 00

No. 2	Proposed	Literature [16]	Literature [17]	Literature [18]
MAE	3.49*E* + 01	3.22*E* + 02	4.02*E* + 02	3.29*E* + 03
MSE	2.71*E* + 04	8.75*E* + 05	4.31*E* + 06	1.44*E* + 07
RMSE	1.65*E* + 02	9.36*E* + 02	2.07*E* + 03	3.80*E* + 03
MAPE	3.20*E* − 03	5.75*E* − 02	2.59*E* − 02	1.59*E* + 00

No. 3	Proposed	Literature [16]	Literature [17]	Literature [18]
MAE	1.43*E* + 02	1.50*E* + 03	1.83*E* + 03	2.89*E* + 03
MSE	2.02*E* + 05	3.25*E* + 07	4.21*E* + 07	3.84*E* + 07
RMSE	4.49*E* + 02	5.70*E* + 03	6.49*E* + 03	6.20*E* + 03
MAPE	2.22*E* − 02	3.85*E* − 02	4.20*E* − 02	6.59*E* − 01

No. 4	Proposed	Literature [16]	Literature [17]	Literature [18]
MAE	2.06*E* + 01	1.32*E* + 02	7.63*E* + 01	2.08*E* + 03
MSE	7.36*E* + 03	7.08*E* + 04	2.14*E* + 04	5.93*E* + 06
RMSE	8.58*E* + 01	2.66*E* + 02	1.46*E* + 02	2.44*E* + 03
MAPE	2.10*E* − 02	4.44*E* − 02	3.31*E* − 02	1.01*E* + 00

No. 5	Proposed	Literature [16]	Literature [17]	Literature [18]
MAE	3.55*E* + 01	1.80*E* + 02	2.23*E* + 02	1.96*E* + 03
MSE	2.98*E* + 04	2.00*E* + 05	7.67*E* + 05	6.48*E* + 06
RMSE	1.73*E* + 02	4.47*E* + 02	8.76*E* + 02	2.55*E* + 03
MAPE	2.80*E* − 03	2.52*E* − 02	2.05*E* − 02	5.35*E* − 01

No. 6	Proposed	Literature [16]	Literature [17]	Literature [18]
MAE	5.61*E* + 01	6.66*E* + 02	4.40*E* + 02	1.86*E* + 03
MSE	2.03*E* + 04	3.65*E* + 06	1.31*E* + 06	6.13*E* + 06
RMSE	1.43*E* + 02	1.91*E* + 03	1.14*E* + 03	2.48*E* + 03
MAPE	1.80*E* − 03	3.30*E* − 02	2.00*E* − 02	7.11*E* − 01

No. 7	Proposed	Literature [16]	Literature [17]	Literature [18]
MAE	1.85*E* + 01	2.79*E* + 02	2.53*E* + 02	1.56*E* + 03
MSE	4.57*E* + 03	6.75*E* + 05	8.77*E* + 05	4.37*E* + 06
RMSE	6.76*E* + 01	8.22*E* + 02	9.36*E* + 02	2.09*E* + 03
MAPE	2.10*E* − 03	2.92*E* − 02	1.96*E* − 02	6.45*E* − 01

No. 8	Proposed	Literature [16]	Literature [17]	Literature [18]
MAE	1.59*E* + 01	1.48*E* + 02	1.12*E* + 02	2.52*E* + 03
MSE	2.71*E* + 03	1.35*E* + 05	7.61*E* + 04	3.26*E* + 07
RMSE	5.21*E* + 01	3.67*E* + 02	2.76*E* + 02	5.71*E* + 03
MAPE	4.30*E* − 03	3.54*E* − 02	2.25*E* − 02	8.38*E* − 01

No. 9	Proposed	Literature [16]	Literature [17]	Literature [18]
MAE	4.02*E* + 01	8.19*E* + 02	9.23*E* + 02	3.56*E* + 03
MSE	2.48*E* + 04	2.42*E* + 07	2.88*E* + 07	2.10*E* + 07
RMSE	1.58*E* + 02	4.92*E* + 03	5.37*E* + 03	4.58*E* + 03
MAPE	2.50*E* − 03	2.24*E* − 02	2.08*E* − 02	1.04*E* + 00

No. 10	Proposed	Literature [16]	Literature [17]	Literature [18]
MAE	2.56*E* + 02	3.80*E* + 02	2.53*E* + 02	3.82*E* + 03
MSE	2.47*E* + 06	1.35*E* + 06	6.03*E* + 05	1.79*E* + 07
RMSE	1.57*E* + 03	1.16*E* + 03	7.76*E* + 02	4.24*E* + 03
MAPE	2.97*E* − 02	6.51*E* − 02	2.53*E* − 02	1.56*E* + 00

## Data Availability

This experiment selects Student-Life and Reach Out online forum post data as the data source. The Student-Life data set is a data set researched by Dartmouth College. The data is open and available.

## References

[1] Grossiord C., Buckley T. N., Cernusak L. A. (2020). Plant responses to rising vapor pressure deficit. *New Phytologist*.

[2] Ma C., Yang Z., Xia R. (2021). Rising water pressure from global crop production-A 26-yr multiscale analysis. *Resources, Conservation and Recycling*.

[3] Schmitt M. T., Neufeld S. D., Mackay C. M. L., Steenbergen O.D. (2020). The perils of explaining climate inaction in terms of psychological barriers. *Journal of Social Issues*.

[4] Spinelli M., Lionetti F., Pastore M., Fasolo M. (2020). Parents’ stress and Children’s psychological problems in families facing the COVID-19 outbreak in Italy. *Frontiers in Psychology*.

[5] Li W., Yang Y., Liu Z. H. (2020). Progression of mental health services during the COVID-19 outbreak in China. *International Journal of Biological Sciences*.

[6] Kotera Y., Laethem M. V., Ohshima R. (2020). Cross-cultural comparison of mental health between Japanese and Dutch workers: relationships with mental health shame, self-compassion, work engagement and motivation. *Cross Cultural & Strategic Management*.

[7] Pei J., Zhong K., Li J. (2021). ECNN: evaluating a cluster-neural network model for city innovation capability. *Neural Computing and Applications*.

[8] Xiang Y.-T., Zhao Y.-J., Liu Z.-H. (2020). The COVID-19 outbreak and psychiatric hospitals in China: managing challenges through mental health service reform. *International Journal of Biological Sciences*.

[9] Holingue C., Kalb L. G., Klein A., Beasley J. B. (2020). Experiences with the mental health service system of family caregivers of individuals with an intellectual/developmental disability referred to START. *Intellectual and Developmental Disabilities*.

[10] Furst M. A., Bagheri N., Salvador-Carulla L. (2021). An ecosystems approach to mental health services research. *BJPsych International*.

[11] Wand T., Buchanan S. H., Derrick K., Harris M. (2020). Are current mental health assessment formats consistent with contemporary thinking and practice?. *International Journal of Mental Health Nursing*.

[12] Areán P. A., Ly K. H., Andersson G. (2016). Mobile technology for mental health assessment. *Dialogues in Clinical Neuroscience*.

[13] Pocobello R., Sehity T., Negrogno L., Minervini C., Guida M., Venerito C. (2020). Comparison of a co‐produced mental health service to traditional services: a co‐produced mixed‐methods cross‐sectional study. *International Journal of Mental Health Nursing*.

[14] Haque A. (2010). Mental health concepts in Southeast Asia: diagnostic considerations and treatment implications. *Psychology Health & Medicine*.

[15] Guo C., Tomson G., Keller C., Soderqvist F. (2018). Prevalence and correlates of positive mental health in Chinese adolescents. *BMC Public Health*.

[16] Papineni K., Roukos S., Ward T., Zhu W. J. Bleu: a method for automatic evaluation of machine translation.

[17] Soet J., Sevig T. (2006). Mental health issues facing a diverse sample of college students: results from the college student mental health survey. *NASPA Journal*.

[18] David E. J. R., Okazaki S., Saw A. (2009). Bicultural self-efficacy among college students: initial scale development and mental health correlates. *Journal of Counseling Psychology*.

[19] Miller K. E., Omidian P., Quraishy A. S. (2006). The Afghan Symptom Checklist: a culturally grounded approach to mental health assessment in a conflict zone. *American Journal of Orthopsychiatry*.

[20] Yang Q., Su Y., Chi C. (2017). Ultrathin graphene-based membrane with precise molecular sieving and ultrafast solvent permeation. *Nature Materials*.

[21] Macaskill A. (2013). The mental health of university students in the United Kingdom. *British Journal of Guidance and Counselling*.

[22] Zhong K., Wang Y., Pei J., Tang S., Han Z. (2021). Super efficiency SBM-DEA and neural network for performance evaluation. *Information Processing & Management*.

[23] Jordan M. I., Mitchell T. M. (2015). Machine learning: trends, perspectives, and prospects. *Science*.

[24] He L., Bai L., Dionysiou D. D. (2021). Applications of computational chemistry, artificial intelligence, and machine learning in aquatic chemistry research. *Chemical Engineering Journal*.

[25] Artrith N., Butler K. T., Coudert F.-X. (2021). Best practices in machine learning for chemistry. *Nature Chemistry*.

[26] Pei J. Solving the problem of charging and discharging of electric vehicles based on particle swarm algorithm.

[27] O’Brien M., Smith C. A., Sokol E. R. (2021). ecocomDP: a flexible data design pattern for ecological community survey data. *Ecological Informatics*.

[28] Zhu Y., Kim M., Zhu X., Kaufer D., Wu G. (2021). Long range early diagnosis of Alzheimer’s disease using longitudinal MR imaging data. *Medical Image Analysis*.

[29] Cobb D. P., Jashami H., Hurwitz D. S. (2021). Bicyclists’ behavioral and physiological responses to varying roadway conditions and bicycle infrastructure. *Transportation Research Part F: Traffic Psychology and Behaviour*.

[30] Liu X., Zhang F., Hou Z. (2021). Self-supervised learning: generative or contrastive. *IEEE Transactions on Knowledge and Data Engineering*.

[31] Wang X., Zhang S., Qing Z. Self-supervised learning for semi-supervised temporal action proposal.

[32] Pei J., Li J., Zhou B., Gao M., Dat Q. A recommendation algorithm about choosing travel means for urban residents in intelligent traffic system.

[33] Rives A., Meier J., Sercu T. (2021). Biological structure and function emerge from scaling unsupervised learning to 250 million protein sequences. *Proceedings of the National Academy of Sciences*.

[34] Abspoel M., Escudero D., Volgushev N. (2021). Secure training of decision trees with continuous attributes. *Proceedings on Privacy Enhancing Technologies*.

[35] Karunadsa P. S., Annakkage U. D., Macdonald B. A. Dynamic security control using secure regions derived from a decision tree technique.

[36] Zhang H., Jiang L., Yu L. (2021). Attribute and instance weighted naive Bayes. *Pattern Recognition*.

[37] Fan J., Zheng J., Wu L., Zhang F. (2021). Estimation of daily maize transpiration using support vector machines, extreme gradient boosting, artificial and deep neural networks models. *Agricultural Water Management*.

[38] Xiao R., Cui X., Qiao H. (2021). Early diagnosis model of Alzheimer’s disease based on sparse logistic regression with the generalized elastic net. *Biomedical Signal Processing and Control*.

[39] Sharma K. K., Seal A. (2021). Spectral embedded generalized mean based k-nearest neighbors clustering with s-distance. *Expert Systems with Applications*.

[40] Sun L., Qin X., Ding W., Xu J., Zhang S. (2021). Density peaks clustering based on k-nearest neighbors and self-recommendation. *International Journal of Machine Learning and Cybernetics*.

[41] Georganos S., Grippa T., Niang Gadiaga A. (2021). Geographical random forests: a spatial extension of the random forest algorithm to address spatial heterogeneity in remote sensing and population modelling. *Geocarto International*.

[42] Brandstätter V., Bernecker K. (2021). Persistence and disengagement in personal goal pursuit. *Annual Review of Psychology*.

[43] Popkov S. I. (2021). Research of interactive and traditional tasks aimed at studying information technologies among students. *Psychological-Educational Studies*.

[44] Ribeiro L. A. C., Bresolin T., Magalhães D. R. G. J., Casagrande D. R., Danes M. A. C., Dórea J. R. R. (2021). Disentangling data dependency using cross-validation strategies to evaluate prediction quality of cattle grazing activities using machine learning algorithms and wearable sensor data. *Journal of Animal Science*.

[45] Tian W., Li Y., Zhou J. (2021). Implantable and biodegradable micro-supercapacitor based on a superassembled three-dimensional network Zn@PPy hybrid electrode. *ACS Applied Materials & Interfaces*.

[46] Zhu W., Ai Y., Fang F., Liao H. (2021). Application of thermosonication in red pitaya juice processing: impacts on native microbiota and quality properties during storage. *Foods*.

[47] Carpenter J. H. (2021). Forty-year natural history study of Bahalana geracei Carpenter, 1981, an anchialine cave-dwelling isopod (Crustacea, Isopoda, Cirolanidae) from San Salvador Island, Bahamas: reproduction, growth, longevity, and population structure. *Subterranean Biology*.

[48] Margolis J. D., Walsh J. P. (2003). Misery loves companies: rethinking social initiatives by business. *Administrative science quarterly*.

